The article "Anti-diabetic, anti-oxidant and anti-hyperlipidemic activities of Melastoma malabathricum Linn. leaves in streptozotocin induced diabetic rats" was retracted in 2023. Reasons: duplicated images; unreliable results or conclusions.

# Anti-diabetic, anti-oxidant and anti-hyperlipidemic activities of *Melastoma malabathricum* Linn. leaves in streptozotocin induced diabetic rats

**DOI:** 10.1186/1472-6882-13-222

**Published:** 2013-09-09

**Authors:** Vikas Kumar, Danish Ahmed, Pushpraj S Gupta, Firoz Anwar, Mohd Mujeeb

**Affiliations:** 1 Department of Pharmaceutical Sciences, Faculty of Health Sciences, Sam Higginbottom Institute of Agriculture, Technology & Sciences (SHIATS)-Deemed University, Allahabad, Uttar Pradesh 211007, India; 2 Sidharatha Institute of Pharmacy, Dehradun, Uttarakhand 248001, India; 3 Department of Photochemistry & Pharmacognosy, Faculty of Pharmacy, Jamia Hamdard, New Delhi 110062, India

**Keywords:** *Melastoma malabathricum*, Streptozotocin, Antidiabetic, Antihyperlipidemic, Glibenclamide

## Abstract

**Background:**

*Melastoma malabathricum* (MM) Linn leaves traditionally use in the treatment of diabetic conditions. The aim of the present investigation was to evaluate the antioxidant, antihyperlipidemic and antidiabetic activity of methanolic extract taken from *Melastoma malabathricum* Linn (Melastomaceae).

**Methods:**

The methanolic leaves extract of MM Linn leaves used for the study. Chemical test of different extract, acute toxicity study and oral glucose test was performed. Diabetes was induced in rat by single intra-peritoneal injection of streptozotocin (55 mg/kg). The rats were divided into following groups: Group I – normal control, Group II (Vehicle) – diabetic control, Group III (STZ-toxic) – MM I (100 mg/kg, p.o.), Group IV – MM II (250 mg/kg, p.o.), Group V – MM III (500 mg/kg, p.o.), Group VI – glibenclamide (10 mg/kg, p.o.). Bodyweight of each rat in the different groups was recorded daily. Biochemical and antioxidant enzyme parameters were determined on day 28. Histology of different organ (heart, liver, kidney, and pancreas) was performed after sacrificing the rats with euthanasia.

**Results:**

The methanolic extract of MM did not show any acute toxicity up-to the dose of 2000 mg/kg and shown better glucose utilization in oral glucose tolerance test. Orally treatment of different doses of MM leaves extract decreased the level of serum glucose, glycated hemoglobin, glucose-6-phosphatase, fructose-1-6-biphosphate and increased the level of plasma insulin, hexokinase. MM treatment decreased liver malondialdehyde but increased the level of superoxide dismutase, catalase and glutathione peroxidase. In oral glucose tolerance test observed increased utilization of glucose. Streptozotocin induced diabetes groups rat treated with different doses of MM leaves extract and glibenclamide significantly increased the body weight. Histopathology analysis on different organ of STZ (streptozotocin) induced diabetic rat show there regenerative effect on the liver, kidney, heart and pancreas.

The article "Anti-diabetic, anti-oxidant and anti-hyperlipidemic activities of Melastoma malabathricum Linn. leaves in streptozotocin induced diabetic rats" was retracted in 2023. Reasons: duplicated images; unreliable results or conclusions.

**Conclusion:**

The antioxidant, antihyperlipidemic and antidiabetic effect of methanolic extract from *Melastoma malabathricum* Linn suggests a potential therapeutic treatment to antidiabetic conditions.

## Background

Diabetes mellitus (DM) is a chronic complication of derangement of protein carbohydrate and lipid metabolism characterized by increased blood glucose level resulting from the defects in insulin secretion insulin action or both [1]. DM is the worldwide problem to leading micro vascular and macrovascular complications [2]. DM is a chronic complication that affected an estimated 135 million people in 1995, 285 million people worldwide in 2010 and data reached approx 500 million people in 2025 mainly increasing in rural and poor population throughout the world [3].

In hyperglycemic condition continuous generation of reactive oxygen species (ROS) occurred. Reactive oxygen species increased the oxidative stress mainly due to over production of oxygen free radicals, as oxidative stress play an important role in development of diabetes. Oxidative stress effect the endogenous antioxidant, which enzyme is responsible for the detoxification of deleterious oxygen radicals [4]. Antioxidant play an important role in the scavenging the free radical, damage the reactive oxygen species and protect the human body from oxidative stress [5]. Hence, drug with both antioxidant and antidiabetic property would be useful for the treatment of the diabetic patient [6]. Medicinal plant is the rich source of various chemical constituent which act on a variety of mechanism to cure the diabetes. Therefore the present study was carried out to evaluate the antioxidant, antihyperlipidemic and antidiabetic effect of *Melastoma malabathricum* Linn leaves.

*Melastoma malabathricum* Linn (MM) is a small shrub from the family Melastomaceae commonly found in tropical and temperate Southeast Asian countries, is locally known to the Malay as Senduduk, India as Phutki. *Melastoma malabathricum* consists of three different varieties, having dark purple-magenta petals flower found in India, other dark purple-magenta petals, light pink-magenta petals and other rare variety having white petals [7]. Generally, different part of the *Melastoma malabathricum* are used in folk medicine to treatment of dysentery, diarrhea, hemorrhoids, leucorrhoea, wounds and cut mainly in India, Malay and Indonesia. Other used infection during confinement and also used to prevent scarring of smallpox and piles [8,9].

Despite long traditional use of *Melastoma malabathricum* leaves in diabetes, no systematic phytochemical and pharmacological work has been carried out on this potential medicinal plant. Therefore the aim of the present study is to find out antioxidant, antihyperlipidemic and antidiabetic effect of *Melastoma malabathricum* (MM) Linn. leaves extract.

The article "Anti-diabetic, anti-oxidant and anti-hyperlipidemic activities of Melastoma malabathricum Linn. leaves in streptozotocin induced diabetic rats" was retracted in 2023. Reasons: duplicated images; unreliable results or conclusions.

## Methods

### Plant materials

Fresh leaves of *Melastoma malabathricum* Linn. was collected in the month of June, 2010 from herbal garden, Department of Life Sciences, Dibrugarh University, Dibrugarh, Assam, India and authenticated by Botanical Survey of India, Shillong, India. A voucher specimen was deposited for future reference.

### Preparation of extracts

The collected leaves of *Melastoma malabathricum* Linn. was washed thoroughly with water to remove the extraporeneous matter. After washing the leaves were dried in shade and grounded 1 kg of powder was extracted with methanol in a Soxhlet apparatus for 3 days. The extract was filtered and the filtrate was concentrated under reduced pressure using a rotatory evaporator at 40°C until the extra solvent completely dried. The yield of methanolic extract was 40%. The extract was stored in the cooling condition in refrigerator at 4°C until further use. The extract was dissolved in 1% carboxyl- methyl cellulose distilled water used for the animal studies.

### Preliminary phytochemical screening of MM extract

The methanolic extract of MM was subjected to preliminary screening for presence of various bioactive pharmaceutical constituents such as glycoside, alkaloids, steroids, protein, flavonoids, tannin, terpenes and saponins [10,11] Table 1.

**Table 1:** **Qualitative phytochemical screening of *Melastoma malabathricum *leaves extract**

**Test name**	**Extracts**					
	**Pet. Ether**	**Benzene**	**Chloroform**	**Acetone**	**Methanol**	**Water**
**Carbohydrates**	**-**	**-**	**-**	**-**	**-**	**-**
**Proteins** &**Amino acids**	**-**	**-**	**-**	**+**	**+**	**+**
**Steroids**	**+**	**+**	**+**	**-**	**-**	**-**
**Saponins**	**-**	**-**	**-**	**-**	**+**	**+**
**Alkaloids**	**-**	**-**	**-**	**-**	**-**	**-**
**Tannins**	**-**	**-**	**-**	**+**	**+**	**+**
**Flavonoids**	**-**	**-**	**-**	**+**	**+**	**+**
**Glycosides**	**-**	**-**	**-**	**-**	**-**	**-**

### Animals

Healthy albino rats (Wistar strain) weight about 170-200 g were kept in individual polyethylene cages and maintained standard condition (12 h dark and 12 h light circle; 25 ± 5°C; 40-60% humidity), and the animals were fed *ad libitum* with normal laboratory chow standard pellet diet, purchased from the Hindustan Liver Limited, Mumbai, India. The animals were allowed to acclimatize for 5 days before commencing the experiments. All the studies were conducted in accordance with the Animal Ethical Committee of Siddhartha Institute of Pharmacy, Dehradun, Uttarakhand (1435/PO/a/11/CPCSEA).

The article "Anti-diabetic, anti-oxidant and anti-hyperlipidemic activities of Melastoma malabathricum Linn. leaves in streptozotocin induced diabetic rats" was retracted in 2023. Reasons: duplicated images; unreliable results or conclusions.

### Acute toxicity studies

For determination of acute toxicity studies the animals were famished overnight and divided into five groups (n = 5). All groups’ animals were fed with different doses of the MM extract in increasing dose level 100, 250, 500, 1000, 2000 mg/kg body weight. The animals were continuously observed for 2 h for the following parameters: [12].

1. Behavioral profile: restlessness, irritability, alertness and fearfulness.

2. Neurological profile: spontaneous activity, touch response, reactivity, pain response and gait.

3. Autonomic profile: urination and defecation.

If any contraindication and death occur after 24 h and 72 h was recorded.

### Oral glucose tolerance test (OGTT)

Oral glucose tolerance test was performed in overnight (16 h) starved normal albino wistar rat. The rats were randomly divided into five groups (n = 6) [13].

Group I rats treated with vehicle only

Group II rats treated with MM extract 100 mg/kg body weight

Group III rats treated with MM extract 250 mg/kg body weight

Group IV rats treated with MM extract 500 mg/kg body weight

Group V rats treated with Glibenclamide 10 mg/kg body weight

Glucose 2 g/kg was fed 30 min after the administration of different doses of MM extract and glibenclamide. Blood was withdrawn from the tail vein at 0, 30, 60, 90 and 120 min, blood glucose level were appraised by the GOD-POD kit (Span diagnostic).

### Induction of diabetes

Diabetes was induced in the overnight fasted male albino wistar rats by a single intraperitoneal injection (i.p.) of streptozotocin (55 mg/kg body weight) dissolved in 0.1 M citrate buffer (pH = 4.5), Normal control rat received citrate buffer only as vehicle. After 3 days induction of diabetes injection of STZ blood sample was collected from the retro-orbital of the rat eyes and plasma, glucose level were determined. The animals confirmed diabetic by the elevated plasma glucose levels (200 mg/dl) were used for the study [14].

### Experiment design

After induction of diabetes animals were divided into six groups of six rats each. Group I: normal control rats administered vehicle only

Group II: diabetic control rats administered tap water only

Group III: tested rats administered MM extract 100 mg/kg body weight

Group IV: tested rats administered MM extract 250 mg/kg body weight

Group V: tested rats administered MM extract 500 mg/kg body weight

Group VI: tested rats administered glibenclamide 10 mg/kg body weight

All group rats received different doses of MM extract and glibenclamide using intragastric tube once daily for 28 days, continuously [15]. According to the acute toxicity testing of the MM extract, the different doses i.e. 100 mg/kg, 250 mg/kg, 500 mg/kg were selected.

The article "Anti-diabetic, anti-oxidant and anti-hyperlipidemic activities of Melastoma malabathricum Linn. leaves in streptozotocin induced diabetic rats" was retracted in 2023. Reasons: duplicated images; unreliable results or conclusions.

### Biological assays

All rats were anesthetized by diethyl ether. The blood samples of each animal were collected from the puncturing retro-orbital plexus and preserved with anticoagulating agents. Blood samples were centrifuged at 4000 rpm at 25°C for 15 min and analyzed for assorted biochemical parameters. The serum total cholesterol, total HDL (High density lipoprotein) cholesterol, total LDL (Low density lipoprotein) cholesterol, and total triglyceride were estimation done spectrophotometrically using standard kits which include serum insulin (Span Diagnostic, India).

### Estimation of antioxidant enzymes

Antioxidant enzyme was estimated by liver homogenate, prepared in ice chilled 10% potassium chloride solution, was used to measure the levels and activities of superoxide dismutase (SOD), catalase (CAT) glutathione peroxidase (GPx) and Malondialdehyde (MDA) by the method [16-18].

### Histopathology

At 28 days all groups animal sacrificed under using mild anesthesia and isolated the different organ (heart, liver, pancreas and liver) of the animal for histopathology. The isolated organ (heart, liver, pancreas and liver) tissue fixed at 40% natural buffered formaldehyde (formalin), dehydrated by passing through a graded series of alcohol, and embedded in paraffin blocks and 5 mm sections were prepared using a semi-automated rotatory microtome. Hematoxylin and eosin were used for staining.

### Statistical analysis

All the data were expressed as the mean ± SEM. and analysis of variance (ANOVA) was used for the statistical analysis using Graph Pad Prism version 5.0 (Software Name is mentioned). The values were considered to be significant when the P value was p < 0.05.

## Results

### Preliminary phytochemical screening

Preliminary phytochemical screening of the methanolic extract of *Melastoma malabathricum* showed terpenoids, flavonoids, phenolic compound, tannins, Saponins, and triterpenes. But the content of flavonoids and phenolic compound were found to be more prominent in the extract (Table 1).

#### Acute toxicity study

An acute toxicity study of the *Melastoma malabathricum* Linn leaves extract were publicized the non-toxic nature of the drug. The different doses of the *Melastoma malabathricum* Linn leaves extract were not showing any toxic reaction or lethality at any of the doses selected until the end of the study period. Acute toxicity of the methanolic extract of *Melastoma malabathricum* revealed the non-toxic nature of the different doses. There were no lethality or toxic reactions found in the selected group which received the different doses of the extract until the end of the experimental period.

The article "Anti-diabetic, anti-oxidant and anti-hyperlipidemic activities of Melastoma malabathricum Linn. leaves in streptozotocin induced diabetic rats" was retracted in 2023. Reasons: duplicated images; unreliable results or conclusions.

#### Effect of MM on oral glucose tolerance test

The acute effect of different doses of MM leaves extract, when administered 30 min, prior to glucose loading produced significant reduction (P < 0.001) in the rise in blood glucose levels, after glucose administration (Table 2). The different doses of MM (100, 250 and 500 mg/kg) produced 11.76%, 19.06% and 31.84% reduction in blood glucose level at 120 min when compared to the vehicle control. Glibenclamide drug was excursion blood glucose level at 26.57% as compared to the vehicle control groups (Figure 1).

**Table 2:** **Effect of *Melastoma malabathricum *leaves extract on oral glucose tolerance test**

**S. no.**	**Groups**	**Time (min)**				
		**0**	**30**	**60**	**90**	**120**
**1**	**Glucose Control**	85.4 ± 2.041	115.4 ± 1.077	112.6 ± 0.0509	106.9 ± 0.872	98.6 ± 0.927
**2**	**Glucose+**	85.8 ± 0.663	105 ± 1.732^*^	101.2 ± 1.655^*^	98.2 ± 0.734^**^	87 ± 1.378^***^
	**MM (100 mg/kg)**					
**3**	**Glucose+**	86.6 ± 0.871	98.2 ± 1.428^*^	94.6 ± 1.077^**^	88.6 ± 1.806^***^	79.8 ± 1.497^***^
	**MM (250 mg/kg)**					
**4**	**Glucose+**	85.8 ± 1.281	89.2 ± 1.655^**^	80.8 ± 1.985^***^	73.6 ± 1.327^***^	67.2 ± 0.861^***^
	**MM (500 mg/kg)**					
**5**	**Glucose+**	84.8 ± 0.583	94.6 ± 1.364^**^	88.4 ± 1.913^***^	81.4 ± 1.435^***^	72.7 ± 0.872^***^
	**Glibenclamide (10 mg/kg)**					

All values represent mean ± SEM *P < 0.05; **P < 0.01; ***P < 0.001; ANOVA, followed by Dunnett’s multiple comparison test.

**Figure 1:** Effect of *Melastoma malabathricum *Linn. (MM) on fasting plasma glucose on oral glucose tolerance test at different concentrations on STZ induced diabetic rats, compared to standard drug Glibenclamide; values are mean ± SEM; n = 6; *P < 0.05; **P < 0.01; ***P < 0.001; P > 0.05 is considered as non-significant (ns).

#### Effect of MM on blood glucose level

The antidiabetic effect of MM leaves extract repeated oral administration on STZ (streptozotocin) induced diabetic rats was presented in Table 3. The administration of different doses (100, 250 and 500 mg/kg) to STZ (streptozotocin) induced diabetic rats caused significantly(P < 0.001) decline the blood glucose level, which was showing that the different doses of MM leaves extract was showing effect at dose dependent manner. Maximum decline rate of blood glucose was observed on day 28 (52.13%, 60.93% and 68.88% respectively). On the other hand glibenclamide showing the 67.26% excursion blood glucose level at compared to the diabetic control groups (Figure 2). MM 500 mg/kg exhibited maximum glucose lowering effect in STZ (streptozotocin) induced diabetic rats compared to the other groups rat received different doses of MM leaves extract and glibenclamide.

The article "Anti-diabetic, anti-oxidant and anti-hyperlipidemic activities of Melastoma malabathricum Linn. leaves in streptozotocin induced diabetic rats" was retracted in 2023. Reasons: duplicated images; unreliable results or conclusions.

**Table 3:** **Effect of *Melastoma malabathricum *leaves extract on blood glucose levels in STZ-induced diabetic rats**

**S. no.**	**Biochemical parameter**	**Normal control**	**STZ-diabetic control**^**a**^	**STZ diabetes+**	**STZ diabetes+**	**STZ diabetes+**	**STZ diabetes+**
				**MM I**^**b**^**(100 mg/kg)**	**MM II**^**b **^**(250 mg/kg)**	**MM III**^**b**^**(500 mg/kg)**	**Glibenclamide**^**b**^**(10 mg/kg)**
**1**	**Fasting plasma glucose (mg/dL)**	81.8 ± 0.969	277 ± 2.608^***^	132.6 ± 1.965^*^	108.2 ± 2.922^**^	86.2 ± 1.428^***^	90.6 ± 0.509^***^
**2**	**Fasting Plasma Insulin (μU/mL)**	14.2 ± 0.583	3.6 ± 0.509^***^	6.8 ± 0.584^*^	10.4 ± 0.601^**^	13 ± 0.316^***^	12.6 ± 0.411^***^
**3**	**Glycated Heamoglobin (A1c) (%)**	1.32 ± 0.073	4.86 ± 0.151^***^	3.72 ± 0.081^*^	2.96 ± 0.678^**^	2.04 ± 0.129^***^	2.16 ± 0.107^***^
**4**	**Hexokinase (μg/mg of tissue)**	147.8 ± 3.484	90.4 ± 3.203^***^	115.6 ± 1.631^*^	131 ± 1.871^**^	142.6 ± 2.015^***^	140.4 ± 2.182^***^
**5**	**Glucose-6-Phosphatase (unit/mg of tissue)**	9 ± 0.707	14.2 ± 0.583^***^	13.4 ± 0.509^*^	11.6 ± 0.611^**^	8.6 ± 0.712^***^	9.8 ± 0.567^***^
**6**	**Fructose-1-6-biphosphatase (unit/mg of tissue)**	28.8 ± 0.861	55 ± 1.012^***^	43.8 ± 1.158^*^	38.2 ± 1.068^**^	30 ± 0.707^***^	31.8 ± 0.861^***^
**7**	**Total Cholesterol (mg/dl)**	78.2 ± 2.011	128 ± 2.366^***^	113.2 ± 2.782^*^	101.4 ± 1.631^**^	87 ± 1.703^***^	89.2 ± 1.393^***^
**8**	**Triglycerides (mg/dl)**	81.4 ± 1.327	134.8 ± 1.356^***^	115.4 ± 1.077^*^	103.6 ± 1.503^**^	90 ± 0.707^***^	93.4 ± 1.077^***^
**9**	**HDL Cholesterol (mg/dL)**	53.2 ± 2.478	28.6 ± 2.441^***^	41 ± 1.732^*^	44.8 ± 1.158^**^	53.8 ± 0.861^***^	52.8 ± 1.655^***^
**10**	**LDL Cholesterol (mg/dL)**	8.92 ± 2.149	72.84 ± 2.812^***^	50.72 ± 3.355^*^	34.08 ± 1.979^**^	15.4 ± 2.302^***^	19.52 ± 1.547^***^
**11**	**VLDL Cholesterol (mg/dL)**	16.28 ± 0.265	26.96 ± 0.271^***^	23.08 ± 0.215^*^	20.72 ± 0.301^**^	18 ± 0.141^***^	18.68 ± 0.215^***^
**12**	**Weight Variation (g)**	192.6 ± 0.872	157.8 ± 1.625^***^	189.4 ± 1.032^***^	186.4 ± 1.749^***^	197 ± 1.304^***^	194.2 ± 1.393^***^

All values represent mean ± SEM *P < 0.05; **P < 0.01; ***P < 0.001; ANOVA, followed by Dunnett’s multiple comparison test.

^a^Compared to vehicle control.

^b^Compared to diabetic control.

**Figure 2:** Effect of *Melastoma malabathricum *Linn. (MM) on fasting plasma glucose at different concentrations on STZ induced diabetic rats, compared to standard drug Glibenclamide; values are mean ± SEM; n = 6; *P < 0.05; **P < 0.01; ***P < 0.001; P > 0.05 is considered as non-significant (ns).

The article "Anti-diabetic, anti-oxidant and anti-hyperlipidemic activities of Melastoma malabathricum Linn. leaves in streptozotocin induced diabetic rats" was retracted in 2023. Reasons: duplicated images; unreliable results or conclusions.

#### Effect of MM of plasma insulin

The effect of different doses of MM leaves extract on plasma insulin was presented in Table 3. In STZ (streptozotocin) induced diabetic rats there is a significant decline in the level of plasma insulin as compared to the normal rat group (rats receiving the vehicle only). Oral administration of different doses of MM leaves extract, significantly (P < 0.001) increased the level of plasma insulin. Amongst all the doses of MM 500 mg/kg was more effective in increasing the level of plasma insulin as compared to other doses of MM and glibenclamide (Figure 3).

**Figure 3:** Effect of *Melastoma malabathricum *Linn. (MM) on level of plasma insulin at different concentrations on STZ induced diabetic rats, compared to standard drug Glibenclamide; values are mean ± SEM; n = 6; *P < 0.05; **P < 0.01; ***P < 0.001; P > 0.05 is considered as non-significant (ns).

#### Effect of MM on glycated haemoglobin (A1c)

The administration of different doses of MM leaves extract was significantly (P < 0.001) increased the level of glycated haemoglobin (A1c) in STZ-induced treated diabetic rats (Table 3). Upon administration of different doses of MM leaves extract (100, 250 and 500 mg/kg) and glibenclamide increased the level of glycated haemoglobin (A1c) in STZ-induced treated diabetic rats to a good extend. The maximum lowering of glycated haemoglobin (A1c) in STZ-induced treated diabetic rats was appeared in group received MM 500 mg/kg dose (Figure 4).

**Figure 4:** Effect of *Melastoma malabathricum *Linn. (MM) on level of glycated hemoglobin (A1c)(%) at different concentrations on STZ induced diabetic rats, compared to standard drug Glibenclamide; values are mean ± SEM; n = 6; *P < 0.05; **P < 0.01; ***P < 0.001; P > 0.05 is considered as non-significant (ns).

#### Effect of MM on hexokinase

The level of hexokinase was observed decrease in STZ treated group rat as compared to the normal group (Table 3). Upon oral administration of different doses of MM leaves extract and glibenclamide were significantly (P < 0.001) boosting the level of hexokinase in STZ-induced treated diabetic rats. STZ (streptozotocin) induced diabetic rats treated with MM leaves extract doses 500 mg/kg showing the maximum increasing the level of hexokinase at compared to the other doses treated group rat (Figure 5).

**Figure 5:** Effect of *Melastoma malabathricum *Linn. (MM) on level of hexokinase (μg/mg of protein) at different concentrations on STZ induced diabetic rats, compared to standard drug Glibenclamide; values are mean ± SEM; n = 6; *P < 0.05; **P < 0.01; ***P < 0.001; P > 0.05 is considered as non-significant (ns).

The article "Anti-diabetic, anti-oxidant and anti-hyperlipidemic activities of Melastoma malabathricum Linn. leaves in streptozotocin induced diabetic rats" was retracted in 2023. Reasons: duplicated images; unreliable results or conclusions.

#### Effect of MM on glucose-6-phosphate

To evaluate the potency of the MM leaves extract on STZ (streptozotocin) induced diabetic rats on glucose-6-phosphate on diabetic rat (Table 3). The level of glucose-6-phosphate was significantly increased in STZ (streptozotocin) induced diabetic groups rat when compared to the normal rat. Upon oral administration of different doses of MM leaves extract and glibenclamide was significantly (P < 0.001) decline the increased level of glucose-6-phosphate. Different doses received groups’ rat significantly decreased the level of glucose-6-phosphate but the dose of MM extract 500 mg/kg was more effective to decline the increased level of glucose-6-phosphate (Figure 6).

**Figure 6:** Effect of *Melastoma malabathricum *Linn. (MM) on level of glucose-6-phosphate at different concentrations on STZ induced diabetic rats, compared to standard drug Glibenclamide; values are mean ± SEM; n = 6; *P < 0.05; **P < 0.01; ***P < 0.001; P > 0.05 is considered as non-significant (ns).

#### Effect of MM on fructose-1-6-biphosphatase

The oral administration of different doses of MM leaves extract and glibenclamide were significantly (P < 0.001) decreases the level of fructose-1-6-biphosphatase in STZ (streptozotocin) induced diabetic rats (Table 3). The level of fructose-1-6-biphosphatase enhance in STZ induced diabetes. STZ (streptozotocin) induced diabetic rats treatment with different doses of MM leaves extract was sharp decrease the level of fructose-1-6-biphosphatase to normalize rat. The MM leaves extract with dose 500 mg/kg shown the supreme diminish levels of fructose-1-6-biphosphatase in comparison to other diabetic treated group rats receiving dose of 100 mg/kg, 250 mg/kg dose of MM and 10 mg/kg of Glibenclamide respectively (Figure 7).

**Figure 7:** Effect of *Melastoma malabathricum *Linn. (MM) on level of fructose-1-6-bisphasphate at different concentrations on STZ induced diabetic rats, compared to standard drug Glibenclamide; values are mean ± SEM; n = 6; *P < 0.05; **P < 0.01; ***P < 0.001; P > 0.05 is considered as non-significant (ns).

#### Effect of MM on lipid profile

To evaluate the effect of MM leaves extract on lipid profile level, the level of cholesterol, triglyceride, LDL (low density cholesterol) and VLDL (very low density cholesterol) were increased and the level of HDL (high density cholesterol) was decreased in the STZ (streptozotocin) induced diabetic rat. Oral administration of MM leaves extract was showed reduction in cholesterol, triglyceride, LDL and VLDL compared to the diabetic control rat group and the level of HDL was increased compared to the diabetic control rat in a significant manner (P < 0.001) (Table 3). MM leaves extract at the doses of 250 mg/kg and 500 mg/kg was more effective than 100 mg/kg in reducing the level of in cholesterol (Figure 8), triglyceride (Figure 9), HDL cholesterol (Figure 10), LDL cholesterol (Figure 11) and VLDL cholesterol (Figure 12) compared to the diabetic control rat.

The article "Anti-diabetic, anti-oxidant and anti-hyperlipidemic activities of Melastoma malabathricum Linn. leaves in streptozotocin induced diabetic rats" was retracted in 2023. Reasons: duplicated images; unreliable results or conclusions.

**Figure 8:** Effect of *Melastoma malabathricum *Linn. (MM) on level of total cholesterol at different concentrations on STZ induced diabetic rats, compared to standard drug Glibenclamide; values are mean ± SEM; n = 6; *P < 0.05; **P < 0.01; ***P < 0.001; P > 0.05 is considered as non-significant (ns).

**Figure 9:** Effect of *Melastoma malabathricum *Linn. (MM) on level of triglyceride at different concentrations on STZ induced diabetic rats, compared to standard drug Glibenclamide; values are mean ± SEM; n = 6; *P < 0.05; **P < 0.01; ***P < 0.001; P > 0.05 is considered as non-significant (ns).

**Figure 10:** Effect of *Melastoma malabathricum *Linn. (MM) on level of HDL cholesterol at different concentrations on STZ induced diabetic rats, compared to standard drug Glibenclamide; values are mean ± SEM; n = 6; *P < 0.05; **P < 0.01; ***P < 0.001; P > 0.05 is considered as non-significant (ns).

**Figure 11:** Effect of *Melastoma malabathricum *Linn. (MM) on level of LDL cholesterol at different concentrations on STZ induced diabetic rats, compared to standard drug Glibenclamide; values are mean ± SEM; n = 6; *P < 0.05; **P < 0.01; ***P < 0.001; P > 0.05 is considered as non-significant (ns).

**Figure 12:** Effect of *Melastoma malabathricum *Linn. (MM) on level of VLDL cholesterol at different concentrations on STZ induced diabetic rats, compared to standard drug Glibenclamide; values are mean ± SEM; n = 6; *P < 0.05; **P < 0.01; ***P < 0.001; P > 0.05 is considered as non-significant (ns).

#### Changes in body weight

Table 3 display the effect of the different doses of MM leaves extract and glibenclamide on the body weight of on the STZ (streptozotocin) induced diabetic rat. At the end of 28 days treatment, the body weight of normal rats, diabetic control, different doses of MM leaves extract and glibenclamide treated rats were observed (Figure 13). Diabetic control group continued to decrease the weight till the end of the study. Glibenclamide and different doses (100, 250 and 500 mg/kg) of MM leaves extract treated rats significantly (P < 0.001) increased the weight as compared to the diabetic control rats.

**Figure 13:** Effect of *Melastoma malabathricum *Linn. (MM) on body weight at different concentrations on STZ induced diabetic rats, compared to standard drug Glibenclamide; values are mean ± SEM; n = 6; *P < 0.05; **P < 0.01; ***P < 0.001; P > 0.05 is considered as non-significant (ns).

The article "Anti-diabetic, anti-oxidant and anti-hyperlipidemic activities of Melastoma malabathricum Linn. leaves in streptozotocin induced diabetic rats" was retracted in 2023. Reasons: duplicated images; unreliable results or conclusions.

#### Effect of MM on antioxidant enzymes

In STZ induced diabetes increase the level of SOD, GPx, CAT and decrease the level of MDA. The level of CAT increased due to increase production of H2O2 in diabetic pancreas and increase the level of SOD due to increased the production of superoxide, which has been implicated in cell dysfunction. The level of antioxidant enzyme SOD (superoxide dismutase), CAT (catalase) and GPx (Glutathione Peroxidase) were significantly (P < 0.001) decreased in diabetic control groups and level of MDA (Malonaldehyde) were significantly increased (Table 4). Glibenclamide (5 mg/kg) and different doses of MM leaves extract (100, 250 and 500 mg/kg) received groups rat signification (p < 0.001) increase the level of SOD (Figure 14), CAT (Figure 15), GPx (Figure 16) and decreased the level of MDA (Figure 17). The result suggests that glibenclamide and all the doses of MM leaves extract increase the level of SOD, CAT and GPx, but MM leaves extract doses 500 mg/kg was more effective in increase the level of SOD, CAT and GPx in diabetic rat as compared with different doses of MM leaves extract and glibenclamide.

**Table 4:** **Effect of *Melastoma malabathricum *leaves extract on antioxidant enzyme at end of the study**

**S. no.**	**Biochemical parameter**	**Normal control**	**STZ-diabetic control**^**a**^	**STZ diabetes+**	**STZ diabetes+**	**STZ diabetes+**	**STZ diabetes+**
				**MM I**^**b**^**(100 mg/kg)**	**MM II**^**b **^**(250 mg/kg)**	**MM III**^**b**^**(500 mg/kg)**	**Glibenclamide**^**b **^**(10 mg/kg)**
**1**	**SOD (U/mg of protein)**	8.6 ± 0.509	3 ± 0.316^***^	4.2 ± 0.374^*^	6.2 ± .432^**^	8 ± 0.323^***^	7.8 ± 0.543^***^
**2**	**CAT (U/mg of protein)**	72.4 ± 1.631	38.6 ± 1.327^***^	46 ± 2.336^*^	56 ± 0.707^**^	68.8 ± 1.158^***^	67.4 ± 1.077^***^
**3**	**GPx (mMH**_**2**_**O**_**2 **_**decomposed/min)**	47 ± 1.183	16.6 ± 0.927^***^	25 ± 0.707^*^	31.6 ± 1.077^**^	42 ± 0.712^***^	40.4 ± 0.927^***^
**4**	**MDA (nmole/mg of protein)**	0.34 ± 0.027	0.66 ± 0.028^***^	0.55 ± 0.017^*^	0.44 ± 0.011^**^	0.36 ± 0.012^***^	0.38 ± 0.016^***^

All values represent mean ± SEM *P < 0.05; **P < 0.01; ***P < 0.001; ANOVA, followed by Dunnett’s multiple comparison test.

^a^Compared to vehicle control.

^b^Compared to diabetic control.

**Figure 14:** Effect of *Melastoma malabathricum *Linn. (MM) on superoxide dismutase (SOD) at different concentrations on STZ induced diabetic rats, compared to standard drug Glibenclamide; values are mean ± SEM; n = 6; *P < 0.05; **P < 0.01; ***P < 0.001; P > 0.05 is considered as non-significant (ns).

The article "Anti-diabetic, anti-oxidant and anti-hyperlipidemic activities of Melastoma malabathricum Linn. leaves in streptozotocin induced diabetic rats" was retracted in 2023. Reasons: duplicated images; unreliable results or conclusions.

**Figure 15:** Effect of *Melastoma malabathricum *Linn. (MM) on Catalase (CAT) at different concentrations on STZ induced diabetic rats, compared to standard drug Glibenclamide; values are mean ± SEM; n = 6; *P < 0.05; **P < 0.01; ***P < 0.001; P > 0.05 is considered as non-significant (ns).

**Figure 16:** Effect of *Melastoma malabathricum *Linn. (MM) on level of Glutathione peroxidase (GPx) at different concentrations on STZ induced diabetic rats, compared to standard drug Glibenclamide; values are mean ± SEM; n = 6; *P < 0.05; **P < 0.01; ***P < 0.001; P > 0.05 is considered as non-significant (ns).

**Figure 17:** Effect of *Melastoma malabathricum *Linn. (MM) on level of Malondialdehyde (MDA) at different concentrations on STZ induced diabetic rats, compared to standard drug Glibenclamide; values are mean ± SEM; n = 6; *P < 0.05; **P < 0.01; ***P < 0.001; P > 0.05 is considered as non-significant (ns).

#### Effect of MM on liver

Liver histopathology studies of STZ induced diabetic rat, the accumulation of fat was increased in the diabetes and large area of hepatocytes taken over by macro droplet of fat. Treatment start with different doses of MM leaves extract as the dose of MM leaves extract increased, the histological condition was improved (Figure 18). The treatment with MM (100 mg/kg) dose shown micro droplet of fat accumulation on rat histopathology, other dose MM (250 mg/kg) dose has shown some micro droplet of fat accumulation on rat liver histopathology as compared to the diabetic control and MM (100 mg/kg) dose. The treatment MM dose (500 mg/kg) shown the rat liver histopathology similar to the glibenclamide drugs (Figure 19).

**Figure 18:** **Effect of *Melastoma malabathricum *Linn. (MM) on liver fat accumulation in different groups of rats: (A) Normal control: (B) Diabetic control: Diabetic control histopathology of rat liver shown the micro fat droplet deposition (yellow arrow) (C) MM I (100 mg/kg): Tested drug histopathology shown granularity and quantity of fat droplet (yellow arrow) were much less compared to the diabetic control. (D)** MM II (250 mg/kg): Tested drug histopathology there was only few micro fat droplet was present (yellow arrow). **(E)** MM III (500 mg/kg): The amount of tested drug increased and the histopathology similar to the glibenclamide treated group. **(F)** Glibenclamide (10 mg/kg): Standard drug treated group shown histopathology similar to the normal control groups. The samples were obtained from the same liver anatomical regions. For each group, 6 rats were examined and 50 pictures were taken. The above picture for each group was chosen randomly from the 80 pictures in this group. Original magnification, 10 ×.

The article "Anti-diabetic, anti-oxidant and anti-hyperlipidemic activities of Melastoma malabathricum Linn. leaves in streptozotocin induced diabetic rats" was retracted in 2023. Reasons: duplicated images; unreliable results or conclusions.

**Figure 19:** **Effect of *Melastoma malabathricum *Linn. (MM) on liver fat accumulation in different groups of rats: (A) Normal control: (B) Diabetic control: Diabetic control histopathology of rat liver had shown the micro fat droplet deposition on round shape (yellow arrow) (C) MM I (100 mg/kg): Tested drug histopathology shown small size of fat droplet (yellow arrow) as compared to the diabetic control. (D)** MM II (250 mg/kg): Tested drug histopathology shown few micro fat droplets (yellow arrow). **(E)** MM III (500 mg/kg): Increased tested drug treated rat histopathology similar to the glibenclamide treated group. **(F)** Glibenclamide (10 mg/kg): Standard drug treated group shown histopathology similar to the normal control groups. The samples were obtained from the same liver anatomical regions. For each group, 6 rats were examined and 50 pictures were taken. The above picture for each group was chosen randomly from the 80 pictures in this group. Original magnification, 40 ×.

#### Effect of MM on heart

Effect of *Melastoma malabathricum* Linn. (MM) on STZ induced diabetic rat heart. In STZ induced diabetes group rat histopathology shown increase the interstitial space increased intercalated disc and increased the level of fat deposition. The treatment starts with dose of MM (100 mg/kg) leaves extract histopathology interstitial space and distort intercalated disc. MM (250 mg/kg) dose histopathology shown less space of interstitial and distort intercalated disc. Increased MM (500 mg/kg) dose treated animal histopathology shown normal histopathology of heart (Figures 20 and 21).

**Figure 20:** **Effect of *Melastoma malabathricum *Linn. (MM) on heart in different groups of rats: (A) Normal control: Normal control group shown normal histopathology of the heart (B) Diabetic control: Diabetic control histopathology shown increased interstitial space and distort the intercalated disc (yellow arrow) (C) MM I (100 mg/kg): Tested drug histopathology shown decreased interstitial space and intercalated disc (yellow arrow) (D) MM II (250 mg/kg): Tested drug histopathology shown less interstitial space (yellow arrow) (E) MM III (500 mg/kg): Tested drug histopathology shown normal heart like the glibenclamide (F) Glibenclamide (10 mg/kg): Glibenclamide treated drug shown the normal histopathology of heart.** The samples were obtained from the same liver anatomical regions. For each group, 6 rats were examined and 50 pictures were taken. The above picture for each group was chosen randomly from the 80 pictures in this group. Original magnification, 10 ×.

**Figure 21:** **Effect of *Melastoma malabathricum *Linn. (MM) on heart in different groups of rats: (A) Normal control: Normal control group shown normal histopathology of the heart there is no changes in interstitial space and intercalated disc. (B) Diabetic control: Diabetic control histopathology shown increased interstitial space, deposition of fats and distort the intercalated disc (yellow arrow) (C) MM I (100 mg/kg): Tested drug histopathology shown decreased interstitial space and having slightly distort intercalated disc (yellow arrow) (D) MM II (250 mg/kg): Tested drug histopathology shown less effect of interstitial space and intercalated disc (yellow arrow) (E) MM III (500 mg/kg): Tested drug histopathology shown normal heart like the glibenclamide (F) Glibenclamide (10 mg/kg): Glibenclamide treated drug shown the normal histopathology of heart.** The samples were obtained from the same liver anatomical regions. For each group, 6 rats were examined and 50 pictures were taken. The above picture for each group was chosen randomly from the 80 pictures in this group. Original magnification, 40 ×.

The article "Anti-diabetic, anti-oxidant and anti-hyperlipidemic activities of Melastoma malabathricum Linn. leaves in streptozotocin induced diabetic rats" was retracted in 2023. Reasons: duplicated images; unreliable results or conclusions.

#### Effect of MM on kidney

STZ induced diabetes in animal histopathology studies of kidney shown inflammation in blood vessels, fat deposition, increase in the thickness of bowman capsules and change in size of the glomerulus. STZ induced diabetic rat treatment with different doses of MM leaves extract improve the injured rat kidney with increasing doses treatment. The treatment with MM (100 mg/kg) dose showed improved kidney histopathology less inflammatory blood vessels, less fat deposition as compared to diabetic control. Treatment with MM (250 mg/kg) dose shown only fat deposition no inflammatory blood vessels and the dose MM (500 mg/kg) shown the normal histopathology there is no inflammatory vessels and no fat deposition (Figures 22 and 23).

**Figure 22:** **Effect of *Melastoma malabathricum *Linn. (MM) on kidney in different groups of rat: (A) Normal control: Normal control histopathology shown 2–5 average size of glomerulus (green arrow) (B) Diabetic control: Diabetic control histopathology shown inflammatory cell in blood vessels (red arrow) and increase the deposition of fats (yellow arrow) (C) MM I (100 mg/kg): Tested drug histopathology shown inflammation in blood vessels (red arrow) and fat deposition (yellow arrow) (D) MM II (250 mg/kg): Tested drug histopathology shown fat deposition (yellow arrow) and increase size of glomerulus (violet arrow) (E) MM III (500 mg/kg): Tested drug histopathology shown normal kidney like the glibenclamide treated group (F) Glibenclamide (10 mg/kg): Glibenclamide treated animal histopathology shown the normal kidney.** The samples were obtained from the same liver anatomical regions. For each group, 6 rats were examined and 50 pictures were taken. The above picture for each group was chosen randomly from the 80 pictures in this group. Original magnification, 10 × .

The article "Anti-diabetic, anti-oxidant and anti-hyperlipidemic activities of Melastoma malabathricum Linn. leaves in streptozotocin induced diabetic rats" was retracted in 2023. Reasons: duplicated images; unreliable results or conclusions.

**Figure 23:** **Effect of *Melastoma malabathricum *Linn. (MM) on kidney in different groups of rat: (A) Normal control: Normal control histopathology shown average size of glomerulus (green arrow) (B) Diabetic control: Diabetic control histopathology shown inflammatory cell in blood vessels (red arrow) and increase the deposition of fats (yellow arrow) (C) MM I (100 mg/kg): Tested drug histopathology shown inflammation in blood vessels (red arrow) and fat deposition (yellow arrow) (D) MM II (250 mg/kg): Tested drug histopathology shown fat deposition (yellow arrow) and increase size of glomerulus (violet arrow) (E) MM III (500 mg/kg): Tested drug histopathology shown normal glomerulus but slightly bigger in size (F) Glibenclamide (10 mg/kg): Glibenclamide treated animal histopathology shown the normal kidney.** The samples were obtained from the same liver anatomical regions. For each group, 6 rats were examined and 50 pictures were taken. The above picture for each group was chosen randomly from the 80 pictures in this group. Original magnification, 40 ×.

#### Effect of MM on pancreas

Histopathology studies of pancreas of STZ induced diabetic rat displayed reduction of the Islets of Langerhans, damaged or reduced the size of β cells and extensive necrosis changes followed by fibrosis and atrophy. STZ induced diabetic rat treated with different doses of MM leaves extract and glibenclamide restored the necrotic and fibrotic changes and raised the number of β cells (Figures 24 and 25).

**Figure 24:** **Photomicrographs of histological changes of rat pancreas of isletes of Langerhans: (A) Normal control: normal histological structure of rat pancreas showing normal islet (green arrow) (B) Diabetic control: diabetic control rat showing dilated acini (blue arrow) and focal necrosis (yellow arrow) (C) MM I (100 mg/kg): tested drug rat showing dilated acini (blue arrow) and focal necrosis (yellow arrow) (D) MM II (250 mg/kg): tested drug rat showing and focal necrosis (yellow arrow) (E) MM III (500 mg/kg): tested drug rat showing and focal necrosis (yellow arrow) (F) Glibenclamide (10 mg/kg): glibenclamide treated rat pancreas showing normal islet (green arrow).** For each group 6 rats were examined and 50 pictures were taken. The above picture for each group was chosen randomly from the 80 pictures in this group. Original magnification, 10 ×.

**Figure 25:** **Photomicrographs of histological changes of rat pancreata (A) Normal control: Normal histological structure of rat pancreata showed averaged sized islet (red arrow) and normal sized β cells (green arrow) (B) Diabetic control: Diabetic control rat showing rat pancreata small sized (red arrow) without enlargement of β cells (yellow arrow) and showing the changes of fatty acid (blue arrow) (C) MM I (100 mg/kg): tested drug rat showing rat pancreata small sized (red arrow) without enlargement of β cells (yellow arrow) and showing the less changes of fatty acid (blue arrow) (D) MM II (250 mg/kg): tested drug rat showing rat showing rat pancreata small sized (red arrow) without enlargement of β cells (yellow arrow) (E) MM III (500 mg/kg): tested drug rat showing rat enlargement of β cells (yellow arrow) (F) Glibenclamide (10 mg/kg): glibenclamide treated rat histological structure of rat pancreata showed averaged sized islet (red arrow) and normal sized β cells (green arrow).** For each group 6 rats were examined and 50 pictures were taken. The above picture for each group was chosen randomly from the 80 pictures in this group. Original magnification, 40 ×.

The article "Anti-diabetic, anti-oxidant and anti-hyperlipidemic activities of Melastoma malabathricum Linn. leaves in streptozotocin induced diabetic rats" was retracted in 2023. Reasons: duplicated images; unreliable results or conclusions.

## Discussion

The present manuscript discuses about the hypoglycemic, antioxidant and Antidiabetic effect of methanolic leaves extract of *Melastoma malabathricum* on normal and streptozotocin (STZ) induced diabetic wistar rats.

Streptozotocin (STZ) is a nitrosourea compound (cytotoxic compound) obtained from soil microbe *Streptomyces achromogenes,* is mediated by reactive oxygen species (ROS). Streptozotocin (STZ) specially penetrates the β-cells via glucose transporter and induce the DNA strand breakage in β-cells causing decrease the endogenous insulin release [19]. The breakage of DNA is due to nitrourea moiety. This breakage of DNA strand leads to amendment the blood sugar level and glucose concentrations in blood. Certain changes start after the administration of Streptozotocin (STZ), two hours after Streptozotocin (STZ) administration, hyperglycemia develops with a concomitant plunge in insulin level [20]. After six hours, hyperglycemia develops with high levels of insulin. Finally, severe hyperglycemia develops with a decrease in insulin levels [21]. In the present investigation the antidiabetic effect of *Melastoma malabathricum* reported first time.

Oral glucose tolerance test is used to identify the altered carbohydrate metabolism during post glucose administration. The ability of methanolic extract of MM to lower the blood glucose level in oral glucose tolerance test suggest that rats treated with different doses of MM extract have better glucose utilization capacity [22]. The results suggest that increased levels of glucose tolerance in different doses of MM extract treated groups were due to insulin emission from β-cells and glucose improved glucose transport and consumption [23].

The article "Anti-diabetic, anti-oxidant and anti-hyperlipidemic activities of Melastoma malabathricum Linn. leaves in streptozotocin induced diabetic rats" was retracted in 2023. Reasons: duplicated images; unreliable results or conclusions.

In Streptozotocin (STZ) induced diabetes groups rat, there is a loss in body weight due to muscle destruction or degradation of structural proteins [24]. Diabetic rats groups received different doses of MM extract and glibenclamide significantly improve the body weight comparison to the diabetic control group rats, all doses of MM extract and glibenclamide showing a protective effect in controlling muscle wasting (reversal of gluconeogenesis). The dose of MM extract (500 mg/kg) showed more improvement in the body weight in comparison to the diabetes control and glibenclamide tested groups.

Glibenclamide persuade insulin secretion from β cell in the pancreas. The leaves extract of MM decreased the serum glucose level and increased pancreatic insulin as shown in our research exertion Therefore result suggests that MM leaves extract may stimulate insulin secretion and decreased serum glucose.

Streptozotocin (STZ) induced diabetes rat decrease the level of plasma insulin. Different doses of MM extract treated groups rat scramble the level of plasma insulin due to active constituent present in the plant extract which persuade insulin secretion or shield the intact function β-cells from further decline so they remain active and continue to produce insulin. The plant extract of MM induces the protection to the β-cells, that result in the decline of blood glucose and diminishes the glucotoxicity to the β-cells [25]. Oral administration of the MM extract for 28 days caused the significant decrease in the blood glucose level with increasing the level of plasma insulin. The possible mechanism of action of MM extract treated groups animal could be potentiating the pancreatic secretion of insulin from β-cells of islets, as was evident by significantly elevating the level of insulin. The hypoglycemic activity of MM extract compared with glibenclamide (standard drug), the results suggest that the mechanism of action of MM extract and glibenclamide may be similar. Insulin is the most important medicine for the treatment of diabetes, a lot of research carried out to find the substitute, secretagogues or sensitizers from synthetic or plant source for the treatment. Some researcher claims that rich source of flavonoids containing plant showed the hypoglycemic and Antidiabetic activity [26,27] and its is reported in our research exertion that *Melastoma malabathricum* leaves extract is the rich source of flavonoids and phenolic compound [28].

STZ induced diabetic rats’ increases the level of lipid peroxidation (MDA), as an indirect evidence of production of free radical [29]. In STZ induced diabetes increase the level of lipid, which cause the development of diabetes and increase the production of free radical formation. Escalating levels of free radical play an important role in causing the hyperglycemia, followed by generation of reactive oxygen species (ROS). Continuous generation of free radicals can lead to tissue damage by attacking membranes through peroxidation of unsaturated fatty acids [30], ROS to elevate the lipid peroxidation and alter the antioxidant defense mechanism and further impair glucose metabolism in biological systems [31,32]. Lipid peroxidation eventually leads to extensive membrane damage and dysfunction [33]. Pancreatic β cell having low level of endogenous antioxidant enzyme and danger to cytotoxic action of free radical. In STZ induced diabetes the level of SOD, GPx, and CAT was increased and the level of MDA was decreased. The level of CAT increased due to increase production of H2O2 in diabetic pancreas and increase the level of SOD due to increased the production of superoxide, which has been implicated in cell dysfunction. Increase the level of SOD without increasing the level of GPx, increase the peroxide level in the cells, cell face the overloading of peroxide. Peroxide can react with transitional metals and generates the radical hydroxyl, which is very harmful radical [34]. On other hand increase the level of superoxide increase the level of GPx, which is directly propositional to MDA (decrease the level of MDA). Different doses of MM extract treated groups significantly improved the level of endogenous antioxidant (SOD, CAT and GPx) and prevent the membrane to damage by decreasing lipid peroxidation compared to diabetic control. Decreased the level of lipid peroxidation (MDA as an indicator) and improved antioxidant status may be one of the mechanism by which drug treatment could contribute to the prevention of diabetic complications [35].

The article "Anti-diabetic, anti-oxidant and anti-hyperlipidemic activities of Melastoma malabathricum Linn. leaves in streptozotocin induced diabetic rats" was retracted in 2023. Reasons: duplicated images; unreliable results or conclusions.

Glycogen plays an important role in the storage of glucose in the form of intracellular storable. Many tissues directly an expression of insulin activity as insulin encourage intracellular glycogen deposition by stimulating glycogen synthesis and inhibiting glycogen phosphorylase. The storage of liver glycogen was markedly reduced in Streptozotocin (STZ) induced diabetes rate, which directly affect the insulin and caused insulin deficiency [36]. Streptozotocin (STZ) induced diabetes rat treated with different doses of MM extract brings back the liver glycogen near the normal rat, which increases the level of insulin secretion.

Streptozotocin (STZ) induced diabetes rat enhanced the level of glycated hemoglobin (A1c) due to excessive production of glucose in blood which further react with blood hemoglobin and prepared the glycated hemoglobin [37]. Three different doses of MM extract were significantly lower the blood glucose, which lead to decreasing the level of glycated hemoglobin. The possible mechanism of action decreasing the blood glucose which is directly propositional to reducing the glycated hemoglobin.

Streptozotocin (STZ) induced diabetes rat escalating the level of total cholesterol and triglyceride. Higher levels of cholesterol (Hypercholesteremia) and higher level of triglyceride (Hypertriglyceridemia) are the primary factor involved in the escalation of coronary heart disease and atherosclerosis, the secondary complications occurring in the diabetes [38]. STZ induced diabetic groups treated with glibenclamide and different doses of MM leaves extract brought back the increased level of total cholesterol and triglyceride near to the normal levels, which could be due to that all drug treated group start the increased level of insulin secretion, which in turn, inhibit hormones sensitive lipase and increase the utilization of glucose and decrease the mobilization of free fatty acids from the fat depositions. STZ induced diabetic groups increased the level of LDL (low density lipoprotein) cholesterol increased the coronary risk factor and decreased level of HDL (high density lipoprotein) cholesterol shown cardiovascular risk factor. In diabetic condition increased the level of TC and TG is associated with increased level of LDL, VLDL and decreased level of HDL. In diabetic condition start the deposition of cholesterol (LDL and VLDL) in peripheral tissue, increased level of LDL and VLDL is atherogenic. Now treatment of the STZ induced diabetes groups start with the different doses of MM leaves extract significantly reducing the serum total cholesterol, triglyceride LDL, VLDL and decreased the level of MDA. The results suggest that different doses of MM extract were significantly lower the blood lipid abnormalities.

Liver is the vital organ and play an important role in defense the postprandial hyperglycemia and synthesis of glucose metabolism. The main role of the liver in glucose utilization is to convert the glucose into glucose-6-phasphatase by the help of hexokinase and other role is it converts glucose into energy [39,40]. STZ induced diabetic groups increased the level of glucose-6-phasphatase, which increase the production of fats to carbohydrates, which turn to deposition into liver, kidney and altered the level of hexokinase, which decreased the conversion and utilization of glucose. Other effect in diabetes is increased the level of fructose-1-6-phasphate. STZ induced diabetic groups treated with different doses of MM leaves extract and glibenclamide increased the level of hexokinase and decrease the level of glucose-6-phasphatase and fructose-1-6-bisphasphate and bring the level near to the normal control.

The article "Anti-diabetic, anti-oxidant and anti-hyperlipidemic activities of Melastoma malabathricum Linn. leaves in streptozotocin induced diabetic rats" was retracted in 2023. Reasons: duplicated images; unreliable results or conclusions.

## Conclusions

Thus, our findings demonstrate that different doses of MM leaves extract has an antidiabetic, antihyperlipidemic and antioxidant effects, which is evidenced by decreased level of blood glucose, glycated hemoglobin, glucose-6-phasphate, fructose-1-6-phasphate, total cholesterol, triglyceride, LDL cholesterol, VLDL cholesterol, SOD, CAT, GPx, and increased level of HDL Cholesterol, plasma insulin, hexokinase, MDA,. Oral glucose tolerance test shown that MM leaves extract having better glucose utilization capacity.

## Competing interests

The authors declare that they have no competing interests.

## Authors’ contributions

VK premeditated and carried out the extraction of the *Melastoma malabathricum*. DA, PSG and MM carried out the biochemical estimations. FA analyses the statistical data and interpretation of histological analysis. All the authors are involved in the critical evaluation of the manuscript. All authors read and approved the final manuscript.

## Pre-publication history

The pre-publication history for this paper can be accessed here:

http://www.biomedcentral.com/1472-6882/13/222/prepub
